The article "Structural and Functional Remodeling of the Brain Vasculature Following Stroke" was published in 2020. Journal: Front Physiol.

# Structural and Functional Remodeling of the Brain Vasculature Following Stroke

**DOI:** 10.3389/fphys.2020.00948

**Published:** 2020-08-07

**Authors:** Moises Freitas-Andrade, Joanna Raman-Nair, Baptiste Lacoste

**Affiliations:** ^1^Neuroscience Program, Ottawa Hospital Research Institute, Ottawa, ON, Canada; ^2^Department of Cellular and Molecular Medicine, Faculty of Medicine, University of Ottawa, Ottawa, ON, Canada; ^3^Brain and Mind Research Institute, University of Ottawa, Ottawa, ON, Canada

**Keywords:** stroke, cerebrovascular, neurovascular unit, vascular remodeling, angiogenesis, blood–brain barrier

## Abstract

Maintenance of cerebral blood vessel integrity and regulation of cerebral blood flow ensure proper brain function. The adult human brain represents only a small portion of the body mass, yet about a quarter of the cardiac output is dedicated to energy consumption by brain cells at rest. Due to a low capacity to store energy, brain health is heavily reliant on a steady supply of oxygen and nutrients from the bloodstream, and is thus particularly vulnerable to stroke. Stroke is a leading cause of disability and mortality worldwide. By transiently or permanently limiting tissue perfusion, stroke alters vascular integrity and function, compromising brain homeostasis and leading to widespread consequences from early-onset motor deficits to long-term cognitive decline. While numerous lines of investigation have been undertaken to develop new pharmacological therapies for stroke, only few advances have been made and most clinical trials have failed. Overall, our understanding of the acute and chronic vascular responses to stroke is insufficient, yet a better comprehension of cerebrovascular remodeling following stroke is an essential prerequisite for developing novel therapeutic options. In this review, we present a comprehensive update on post-stroke cerebrovascular remodeling, an important and growing field in neuroscience, by discussing cellular and molecular mechanisms involved, sex differences, limitations of preclinical research design and future directions.

## General Concepts

Stroke is an injury to the central nervous system (CNS) with a vascular cause, leading to high rates of disability and representing the second leading cause of death worldwide (Mittmann et al., 2012; Krueger et al., 2015; Mozaffarian et al., 2015). Stroke compromises cerebral blood flow (CBF) following either blood vessel occlusion (i.e., *ischemic stroke*) or blood vessel rupture (i.e., *hemorrhagic stroke*), which includes intracerebral hemorrhage (ICH) or subarachnoid hemorrhage (SAH) (Sacco et al., 2013). Hemorrhagic strokes represent ∼20% of cases, while ischemic lesions account for almost 80% of all strokes (Qureshi et al., 2009; Donkor, 2018). Most stroke survivors are left with residual impairments requiring chronic rehabilitation therapy (Bernhardt et al., 2019; Hayward et al., 2019). Moreover, the 30-day mortality rate of ischemic stroke has been estimated at ∼15% in high-income countries (Gattringer et al., 2019), which may vary depending on sex-specific factors (Arnao et al., 2016) and economic disparities (Osypuk et al., 2017). A recent study from the Netherlands showed that in >15,000 patients who had a first stroke at age 18–49 in 1998–2010, cumulative 15-year mortality among 30-day survivors was 13.3 per 1,000 person-years, compared with an expected mortality of 2.4 per 1,000 person-years in the general population (Ekker et al., 2019). In addition, brain microinfarcts (<5 mm lesions) play an insidious role in aging and dementia, since these microscopic strokes may accumulate over several years before manifesting as detectable symptoms (Hakim, 2014; Ferro et al., 2019).

By limiting tissue perfusion, stroke affects both neuronal health and vascular health (Iadecola and Anrather, 2011a, b; Tymianski, 2011; Silasi and Murphy, 2014) with widespread consequences. While numerous lines of investigation have aimed to develop neuroprotective therapies for stroke (Dirnagl et al., 2013; Willis and Hakim, 2013; Corbett et al., 2014; Meschia et al., 2014; Ploughman et al., 2015), there were too few significant advances. For instance, only thrombolysis with recombinant tissue plasminogen activator rtPA (Hebert et al., 2016) or acute endovascular treatment (Goyal et al., 2015) have led to significant benefit for ischemic stroke (Richardson et al., 2014; Teasell et al., 2014a, b; Gurewich, 2016). Within the first hours after ischemic stroke, the goal is to promptly restore perfusion (Lin and Sanossian, 2015; Prabhakaran et al., 2015), and intravenous administration of rtPA has been the first line of intervention for years (The National Institute of Neurological Disorders, and Stroke rt-Pa Stroke Study Group, 1995; Gurewich, 2016). Unfortunately, rtPA must be administered within a narrow therapeutic window (∼4 h following stroke). Moreover, due to safety concerns, its use is limited to 10–15% of stroke victims (Jauch et al., 2013; Gurewich, 2016; Suzuki et al., 2016).

Maintenance of brain health is ensured by key vascular features: (i) The safeguarding of vascular networks for efficient perfusion; (ii) The function of the blood–brain barrier (BBB) to preserve brain homeostasis; and (iii) The regulation of CBF to match energy demands of brain cells (Andreone et al., 2015). During development, neuronal and vascular network formation share similar mechanisms of growth and maturation (Carmeliet and Tessier-Lavigne, 2005; Gu et al., 2005; Eichmann and Thomas, 2013). Endothelial cells (ECs) secrete factors that modulate neurogenesis (Goldman and Chen, 2011; Delgado et al., 2014; Licht and Keshet, 2015; Walchli et al., 2015) and neuronal activity controls brain angiogenesis and barriergenesis (Lacoste, 2014; Biswas et al., 2020). In the mature brain, relationships between neural and vascular cells ensure a functional matching such that changes in neuronal activity are coupled to changes in CBF (i.e., neurovascular coupling) (Hillman, 2014). This involves balanced secretions of vasoconstrictor and vasodilator molecules including, but not limited to, endothelial-derived nitric oxide (NO), or astrocyte-derived prostaglandin E_2_ (PGE_2_) (Attwell et al., 2010; Cauli and Hamel, 2010; Mishra et al., 2016). The underlying structure of neurovascular coupling is the neurovascular unit (NVU), which corresponds to a multicellular ensemble in which ECs, neurons, pericytes, astrocytes, and microglia orchestrate brain function (Zlokovic, 2010; Lind et al., 2013; ElAli et al., 2014; Howarth, 2014) (Figure 1). The NVU also constitutes the BBB which controls the efflux/influx of substances for a controlled brain homeostasis (Daneman, 2012; Ben-Zvi et al., 2014; Andreone et al., 2015; Profaci et al., 2020). The structural and functional interdependence between brain cells and blood vessels renders the brain particularly vulnerable to declines in CBF that result from stroke.

**FIGURE 1:** Cellular and acellular constituents of the neurovascular unit (NVU). **(A)** At the level of penetrating arteries, upstream capillaries, endothelial cells (ECs) are surrounded by vascular smooth muscle cells. At this level, cerebral vessels are still surrounded by the pia. The Virchow–Robin space is located between the pia and the glial limitans formed by the astrocytic endfeet. This perivascular space plays an important role in waste removal and in regulation of the interstitial fluid of the brain. **(B)** At the level of intracerebral capillaries, the NVU is comprised of ECs, pericytes, astrocytes, microglia, and the basement membrane. Both the ECs and surrounding pericytes are unsheathed by a common basement membrane. Pericyte processes encase most of the endothelial surface. Astrocytic endfeet completely surround the capillary wall. Resting microglial have a ramified morphology and are in constant surveillance around brain microvessels. Gap junction channels enable cytoplasmic continuity between astrocytic endfeet, and also exist between pericytes and ECs at peg-socket structures providing quick communication between these cells. Specialized tight junctions between ECs prevent paracellular leakage into the brain parenchyma. **(C)** The NVU undergoes dramatic structural changes following stroke, affecting cerebrovascular integrity, neuro-vascular coupling and neuronal survival within the peri-infarct territory. *Figure prepared with BioRender.*

Post-stroke NVU remodeling represents a growing field in neuropathophysiology (Maki et al., 2013; Knowland et al., 2014; Liu et al., 2014; Prakash and Carmichael, 2015; Munji et al., 2019). While the mechanisms underlying ischemia-induced neuronal plasticity are an ongoing focus in stroke research (Mostany et al., 2010; Swayne and Wicki-Stordeur, 2012; Silasi and Murphy, 2014; Felling and Song, 2015), our understanding of acute and chronic vascular responses to stroke is only in its infancy. NVU remodeling is rapidly activated after stroke and occurs at the molecular and cellular levels. Within minutes following an ischemic insult, proangiogenic genes are upregulated and growth factors are secreted to promote both angiogenesis and survival of glial and neuronal cells within peri-infarct tissues (Ergul et al., 2012; Gutierrez-Fernandez et al., 2012; Talwar and Srivastava, 2014). These events stimulate neurogenesis, synaptogenesis and neuronal plasticity, improving functional outcome (Ergul et al., 2012). In addition, changes in mechanical shear stress due to arterial occlusion result in increased flow through pre-existing collaterals and trigger significant changes in blood vessels (Nishijima et al., 2015). Paradoxically, endogenous repair mechanisms also have detrimental effects on the brain vasculature, as we will discuss in this review. Altogether, these cellular and molecular responses to stroke contribute to vascular and neuronal injury (Haley and Lawrence, 2016; Nahirney et al., 2016).

Despite recent advances in significant areas of stroke pathophysiology, certain aspects of stroke, and particularly spatiotemporal cerebrovascular responses, require further attention. Stroke doubles the risk for dementia (post-stroke dementia), and approximately 30% of stroke survivors develop cognitive dysfunction within 3 years (Allan et al., 2011; Vijayan and Reddy, 2016). The link between stroke and dementia was also observed in patients younger than 50 years, up to 50% of whom exhibit cognitive deficits after a decade (Schaapsmeerders et al., 2013). There is also mounting evidence indicating that stroke can precipitate the likelihood of developing neurodegeneration (Vijayan and Reddy, 2016). Vascular vulnerabilities caused by stroke result in neurovascular uncoupling and affect the integrity of the BBB; these changes impact proper brain functioning and are characteristics found in the early stages of several neurological disorders including Alzheimer’s disease. Therefore, understanding the mechanisms involved in cerebrovascular adaptation to brain injury may have profound long-term clinical outcomes. In this review, we present an overview of recent advances in cerebrovascular research on stroke, and we discuss limitations and ideas for future investigation.

## Effects of Stroke on the Neurovascular Unit

Capillary brain ECs and surrounding pericytes, astrocytes, microglia, neurons, and extracellular matrix (ECM) of the basement membrane altogether compose the NVU. The multiple interactions between these cellular and acellular elements are disrupted after stroke.

### Effects of Stroke on Endothelial Cells

#### Effects of Stroke on Endothelial Cell Structure and Molecular Profile

The EC layer provides the CNS with an important physical, functional, and metabolic barrier, which limits the entry of circulating hydrophilic molecules, such as peptides and proteins into the brain parenchyma. Gaseous molecules such as oxygen (O_2_) and carbon dioxide (CO_2_), as well as small lipophilic molecules less than 500 Da can diffuse freely through brain ECs. Brain ECs are attached to each other by specialized ‘tight’ junctions (TJs) consisting of various molecular components (Chow and Gu, 2015; Delaney and Campbell, 2017). The TJs form the physical barrier of the BBB (Reese and Karnovsky, 1967) and regulate permeability of the endothelial layer. TJ proteins have also been implicated in regulation of gene expression, cell proliferation and differentiation (Zlokovic, 2008; Sweeney et al., 2019). Brain ECs also express gap junction proteins, such as connexin (Cx)-37, Cx40 and Cx43 that contribute to TJ integrity (Nagasawa et al., 2006; De Bock et al., 2011) and cell–cell communication (Figueroa and Duling, 2009; De Bock et al., 2014). The role of endothelial Cxs in BBB function, particularly during aging, remains poorly explored (De Bock et al., 2014).

TJ disruption is a hallmark of both ischemic and hemorrhagic stroke and is typically associated with increased vascular permeability and homeostatic changes in the neuronal microenvironment. It was shown in an ischemia/reperfusion model that BBB permeability exhibited a biphasic pattern (permeability occurring at 3 and 72 h of reperfusion), which was linked to changes in claudin-5, occludin and ZO-1 protein levels (Jiao et al., 2011). More recently, Knowland et al. (2014) used transgenic mice expressing a fusion protein of eGFP with claudin-5 and elegantly demonstrated that TJs were stable during the early phase of reperfusion (up to 24 h) following 30 min of transient middle cerebral artery occlusion (tMCAo), but underwent significant remodeling and breakdown from 48 to 58 h after reperfusion (Knowland et al., 2014). This study demonstrates the stepwise dysfunction that occurs initially at the transcellular level followed by paracellular impairment that accounts for BBB deficits in stroke. Furthermore, it links caveolin-1 (cav-1) to impaired transcellular route.

Caveolae-mediated transcytosis is a major pathway for transport across ECs and it is normally suppressed in the healthy brain (Drab et al., 2001; Predescu et al., 2001; Schnitzer, 2001; Tuma and Hubbard, 2003; Ben-Zvi et al., 2014). Caveolae are 50–100 nm invaginations in the plasma membrane and are highly enriched in saturated phospholipids, sphingolipids, ethanolamine plasmalogens and cholesterol (Andreone et al., 2017). The formation of caveolae vesicles requires both caveolin coat proteins and cytosolic adaptor proteins belonging to the cavin family (Ayloo and Gu, 2019). Under physiological conditions, major facilitator super family domain containing 2a (MFSD2A) is selectively expressed in brain endothelium (Ben-Zvi et al., 2014). MFSD2A acts as a lipid flippase, transporting phospholipids, from the outer to inner plasma membrane leaflet thus altering the plasma membrane composition in such a way that caveolae vesicles are unable to form (Andreone et al., 2017). Inhibition of caveolae formation and trafficking ensures BBB integrity under normal conditions. However, caveolae-mediated transcytosis is activated following tMCAo, and cav-1 expression increases early following stroke or brain injury, prior to TJ disassembly (Knowland et al., 2014). A significant correlation between the extent of BBB disruption following brain ischemia and cav-1 expression was recently confirmed in mice subjected to focal cortical ischemia induced by photothrombosis (Choi et al., 2016). In summary, ischemia/reperfusion-induced BBB disruption in the peri-infarct region involves (i) upregulation of caveolae-mediated endothelial transcytosis in the early phase of reperfusion (between 0 and 12 h); (ii) major TJ remodeling in the late phase (48–60 h) (Cipolla et al., 2004; Knowland et al., 2014; Haley and Lawrence, 2016; Nahirney et al., 2016). The first phase, which peaks at 6 h, leads to non-selective vesicular transport of blood-borne molecules across ECs. The second phase leads to breakdown of the vessel wall, exacerbating BBB dysfunction. It remains unclear why ECs respond in two phases and whether increased transcytosis provides a signal to the NVU. An enticing notion would be to test whether stroke disrupts the unique endothelial cell membrane lipid composition in such a way that induces cav-1 dependent transcytosis. Other factors can also be at play, for example, in a mouse model of retinal vein occlusion, activated ECs expressed caspase-9, the caspase-9 induced non-apoptotic endothelial dysfunction, and barrier breakdown (Avrutsky et al., 2020). Nonetheless, BBB disruption via increased caveolae-mediated bulk-flow fluid transcytosis allows free mobility of toxic substances and accumulation into the brain of plasma proteins that notably include immunoglobulins, albumin, laminin, thrombin and ferritin, collectively leading to neuroinflammation, neuronal death and functional impairment (Zlokovic, 2010).

Other important endothelial players are involved in vascular responses to stroke. Rho-associated coiled-coil kinase (ROCK), a downstream effector of the small GTPase RhoA, is a major regulator of endothelial function (van Nieuw Amerongen et al., 2003; Allen et al., 2010; Mikelis et al., 2015; De Silva et al., 2016) and is involved in the pathogenesis of vascular diseases (Yao et al., 2010; Hartmann et al., 2015; Kajikawa et al., 2015). ROCKs belong to the serine-threonine family of kinases, with two isoforms (1 and 2) that play different pathophysiological roles (Hartmann et al., 2015). Both ROCK1 and ROCK2 are expressed in ECs (Montalvo et al., 2013), and ROCK2 is abundantly found in the brain (Nakagawa et al., 1996) where it plays a pivotal role in endothelial homeostasis. ROCKs play integral roles in cell adhesion, migration and proliferation (Riento and Ridley, 2003) and when activated by RhoA it regulates assembly of the actin cytoskeleton and smooth muscle cell contractility (Noma et al., 2012). In rodent tMCAo, ischemia-reperfusion promotes RhoA/ROCK signaling (Cui et al., 2013; Canazza et al., 2014). Pathological RhoA/ROCK2 activation in ECs promotes the association between endothelial NO synthase (eNOS) and cav-1 and their translocation to membrane caveolae compartments (Zhu et al., 2003) where eNOS is inhibited (Ju et al., 1997; Drab et al., 2001; Ming et al., 2002), which might in turn impair permeability (Siddiqui et al., 2011). *In vivo* evidence from pharmacological studies in mice show that non-selective inhibition of ROCKs following tMCAo exerts neurovascular protection by significantly reducing lesion volumes and improving CBF, in an endothelium-dependent manner (Rikitake et al., 2005; Shin et al., 2007; Sugimoto et al., 2007; Satoh et al., 2010; Vesterinen et al., 2013). Non-selective inhibition of ROCKs by hydroxyfasudil also attenuates early BBB disruption following intracerebral hemorrhage in rats (Fujii et al., 2012; Fu et al., 2014). Selective pharmacological ROCK2 inhibition by KD025 (SLx-2119) was recently demonstrated as efficacious and safe acutely after tMCAo in mice (Lee et al., 2014). ROCK also directly inhibits expression of eNOS (*Nos3*) by decreasing the mRNA stability of eNOS (Noma et al., 2012). Interestingly, expression and activity of eNOS are constitutively enhanced in brain ECs from heterozygous ROCK2 knockout (*Rock2*^+/–^) mice that display reduced infarct volume following tMCAo (Hiroi et al., 2018). Accumulating *in vitro* evidence also shows that increased expression and activity of ROCKs in ECs account for ischemia-induced barrier dysfunction, for instance following oxygen-glucose deprivation (OGD) (Allen et al., 2010; Gibson et al., 2014; Yang et al., 2016). Pathological activation of ROCK2 also promotes oxidative stress (Rivera et al., 2007; Soliman et al., 2012), and pharmacological blockade of ROCKs reduces OGD-induced hyperpermeability via inhibition of endothelial oxidative stress (Gibson et al., 2014).

As a result of a tightly sealed BBB, brain ECs express specialized transporter proteins on both their luminal and abluminal surfaces. Efflux transporters, primarily localized on the luminal surface, include ATP-binding cassette (ABC) transporters, the multidrug resistance transporter P-glycoprotein (Pgp) and several multidrug resistance-associated proteins (MRPs) that work together to reduce penetration of toxic compounds into the brain (Shen and Zhang, 2010). Among many other transport systems, brain ECs also express the glucose transporter-1 (GLUT1), involved in delivering glucose into the brain (Winkler et al., 2015; Tang M. et al., 2017; Vaudano et al., 2017). For instance, isolated bovine brain capillaries subjected to an OGD paradigm displayed decreased Pgp and MRP expression after 24 h of reoxygenation (Tornabene et al., 2019). Interestingly, vitamin E α-tocotrienol was reported as protective against tMCAo in mice through upregulation of MRP-1, resulting in an increase in efflux of toxic oxidized glutathione (Park et al., 2011). In this study, the authors investigated the effects of α-tocotrienol on neuronal MRP-1, but the role of endothelial MRP-1 in the context of ischemia/reperfusion remains to be explored.

Cerebral ECs also express a wide array of ion transporters and channels, asymmetrically distributed between the luminal and abluminal plasma membranes. This polarized arrangement of channels and transporters allows ECs to participate in the regulation of brain interstitial fluid volume and composition. During the early hours following ischemic stroke in animal models, edema builds up via processes involving stimulation of EC ion transporters on the luminal side and increased secretion of Na^+^, Cl^–^, followed by water from the blood stream into the brain across the BBB (O’Donnell, 2014). These transporters also represent possible targets for therapeutic intervention in stroke (O’Donnell, 2014; Brzica et al., 2017).

As mentioned earlier, endogenous mechanisms recruited following brain ischemia have detrimental effects on the brain vasculature (Beck and Plate, 2009). Vascular endothelial growth factor (VEGF) is a potent inducer of microvascular permeability (Dvorak, 1995; Zhang et al., 2002) via rapid (within minutes) stimulation of caveolae-mediated transcytosis (Feng et al., 1999; Chen et al., 2002). Moreover, oxidative stress is promptly elevated in the peri-infarct region (Carbonell and Rama, 2007; Shi and Liu, 2007; Pradeep et al., 2012; Rodrigo et al., 2013) and represents a major cause of vascular dysfunction through neutralization of NO by reactive oxygen species. This decreases NO bioavailability and inhibition of its modulatory role in angiogenesis and vascular reactivity (Nedeljkovic et al., 2003; Park et al., 2005; Fisher, 2008; Xu C. et al., 2016; van Leeuwen et al., 2020). Interestingly, in patients with acute stroke, low NO levels following stroke correlate with outcome severity (Rashid et al., 2003). Oxidative stress also induces vascular hyperpermeability through oxidant-induced phosphorylation of cav-1 and increased caveolae-mediated transcytosis in ECs in culture (Takeuchi et al., 2013). Altogether, these mechanisms contribute to the early-onset vascular injury observed in the peri-infarct region (Haley and Lawrence, 2016; Nahirney et al., 2016).

Collectively, these studies reveal a high complexity at the level of the BBB, which raises challenges but also new opportunities for stroke therapy (Abdullahi et al., 2018; Liberale et al., 2020). Recent publications are unmasking novel endothelial metabolic pathways that are conserved across diseases and species (Rohlenova et al., 2020). Interestingly, Munji et al. (2019) recently investigated brain EC transcriptomic changes in four different brain injury models associated with BBB disruption: permanent MCAo (coagulation of the distal portion of the left middle cerebral artery), experimental encephalomyelitis, traumatic brain injury and kainate-induced seizures (Munji et al., 2019). Remarkably, 2 days following injury onset, when the most severe BBB dysfunction was observed, 54 common genes were upregulated in all four injury models, and 136 genes appeared upregulated in at least three models. These include genes that regulate leukocyte trafficking and proteolytic cleavage of ECM. Multiple members of several gene families were upregulated: extracellular proteases of the Serpin family (Serpine1 and Serping1), Adams and Adamts families (Adam12, Adam19, Adamts4, and Adamts8), collagens (Col1a1, Col1a2, Col3a1, Col5a1, Col5a2, and Col12a1), centromere proteins (Cenpe and Cenpf), Igf-binding proteins (Igfbp4 and Igfbp5), kinesins (Kif11, Kif15, and Kif20b), lysyl oxidases (lox, Loxl2, and Lox3), sulfatases (Sulf1 and Sulf2), thrombospondins (Thbs1 and Thbs2), and pleckstrin domain-containing genes (Plekho1 and Plekho2). Taken together, BBB dysfunction-induced changes in gene expression affect cell division, blood vessel development, inflammatory response, wound healing, leukocyte migration and focal adhesion, highlighting a role for angiogenesis and inflammation in this response (Munji et al., 2019). In addition, mesenchyme homeobox 1 (Meox1), placental growth factor (pgf) and insulin-like growth factor binding protein 4 and 5 (Igfpb4 and 5) were among the genes associated with angiogenesis and upregulated following stroke (Freitas-Andrade et al., 2012; Smith et al., 2018; Wu et al., 2018; Munji et al., 2019). The authors also found that, in each disease model, brain ECs acquired a “peripheral” (i.e., leakier) endothelial gene expression profile. These findings highlight the importance of transcriptomic studies that reveal novel pathways involved in brain endothelial dysfunction and unmask common pathways that may be significant targets for stroke therapy. Of note, while this elegant study provides invaluable molecular insights into BBB dysfunction, the animals used for MCAo were all young, 2–3-month-old males (Munji et al., 2019). Limitations related to the age of animal models are discussed later in this review.

#### Effects of Stroke on Endothelial Cell Function

Endothelial cells are master regulators of neurovascular coupling and CBF (defined as the blood volume that flows per unit mass or volume of brain tissue per time unit) in the healthy brain, in particular through production of vasodilatory NO via eNOS (Yamada et al., 2000). However, other factors produced by ECs such as, epoxyeicosatetraenoic acids (EETs), prostacyclin as well as endothelium-derived hyperpolarizing factor (EDHF) can also trigger vasodilation (Kisler et al., 2017). For example, mechanical shear stress in vessel lumen activates EC production of arachidonic acid (AA) and its metabolic products EETs via cytochrome P450 activity, and prostacyclin via cyclooxygenase 1 (COX1) activity. These by-products act on the surrounding vascular smooth muscle cells (VSMCs) and induce vasodilation (Kisler et al., 2017). Under pathological conditions, dysregulation of eNOS activity is involved in cardiovascular disease, vascular aging, vascular dementia and stroke (Huang et al., 1995; Lange-Asschenfeldt and Kojda, 2008; Sawada and Liao, 2009; Toda et al., 2009; Toda, 2012; Zhu et al., 2016; Wang et al., 2018). eNOS is constitutively expressed in ECs, briefly activated by increases in intracellular calcium, and underlies agonist (e.g., acetylcholine)-induced endothelium-dependent vasodilation. NO released by ECs triggers relaxation of VSMCs, and a partial modulation of eNOS is sufficient to induce large changes in CBF (Samdani et al., 1997).

Ischemic stroke, resulting in acute loss of regional CBF, rapidly initiates vascular remodeling via eNOS (Liu et al., 2014; Hoffmann et al., 2015; Lapi and Colantuoni, 2015; Prakash and Carmichael, 2015). Following MCAo in rats, while eNOS inhibitors reduce CBF and increase infarct volume, intra-arterial administration of NO donors increases CBF and decreases infarct volume (Dalkara and Moskowitz, 1994; Dawson, 1994; Iadecola, 1997). As such, eNOS activation is considered neuroprotective (Zhu et al., 2016). The Statin class of drugs, which upregulate eNOS, have neuroprotective properties in experimental animal models of stroke (Vaughan and Delanty, 1999). The upregulation of eNOS by Statins is mediated by inhibition of small GTPase RhoA (Sawada and Liao, 2009), reducing activation of RhoA’s downstream effector ROCK2 (Hao et al., 2016; Tang F. C. et al., 2017). Using pharmacological intervention to directly target eNOS function might represent an interesting avenue to promote stroke recovery. This is important as direct eNOS modulation may prevent expansion of penumbral cell death, a notorious clinical problem. The effects of eNOS enhancers on stroke recovery have not yet been tested in animal models of stroke. AVE3085 and AVE9488 are small-molecule eNOS enhancers that are protective in rodent models of cardiovascular disease, including heart failure, myocardial infarction and diabetes (Bauersachs and Widder, 2008; Fraccarollo et al., 2008; Wohlfart et al., 2008; Frantz et al., 2009; Schafer et al., 2009; Cheang et al., 2011). These therapeutic benefits were attributed to ameliorated endothelial function via increased NO bioavailability and reduced oxidative stress.

In the cerebral vasculature, direct intercellular communication through gap junctions is instrumental, as synchronization of VSMCs and ECs along the vessel is required for proper vasomotor tone. Indeed, the low electrical resistance of these channels allows for faster signaling over long distances such as retrograde propagation of dilation to upstream arteries; gap junctions are hence critical in conducting a hyperpolarizing, electrical wave between ECs that modulates vascular tone (Behringer and Segal, 2012). Gap junction communication between the endothelium and astrocytes, as well as between ECs and pericytes, mediate neurovascular coupling and vasomotor control, respectively (De Bock et al., 2017; Pohl, 2020). For example, several endothelial signaling factors that control vasomotor function, such as prostacyclin and NO, rely on the increase in endothelial intracellular Ca^2+^ concentration. Gap junctional transfer of Ca^2+^ (or Ca^2+^ releasing compounds) plays an important role in controlling endothelial-dependent vasomotor function (Pohl, 2020). Under stroke conditions, this finely tuned coupling between cells is disrupted (Bolon et al., 2005; Yu et al., 2010). The role of endothelial gap junctions in CBF after stroke remains to be fully elucidated.

Collateral vascular remodeling, a process known as arteriogenesis, is initiated by fluid shear stress rather than hypoxia (Nishijima et al., 2015). ECs lining the collateral vasculature detect increased flow shear stress, which triggers the expression of transient receptor potential cation channel, subfamily V, member 4 (Trpv4) (Schierling et al., 2011). This mechanosensitive Ca^2+^ channel has been shown to induce significant collateral growth length and diameter in rats subjected to bilateral common carotid artery occlusion. Indeed, proper collateral vascular responses in stroke can significantly affect stroke outcome and mortality (Kimmel et al., 2019; Nannoni et al., 2019). However, current understanding of collateral vessel dynamics is not clear; interestingly, a recent study reported that collateral vessels have distinct endothelial and smooth muscle cell phenotypes (Zhang et al., 2019). Understanding the molecular factors that govern collateral responses to brain injury may illuminate new avenues for therapeutic approaches.

### Effects of Stroke on Pericytes

#### Effects of Stroke on Pericyte Structure

Pericytes are cells located within the basement membrane surrounding cerebral capillaries, and are in intimate contact with ECs through gap junctional complexes, called peg-socket contacts where the basement membrane is absent (Figure 1B). Pericytes represent a heterogeneous cell population with differences in morphology, location within the vascular tree and function (Winkler et al., 2014). Pericyte subtypes include ‘mid-capillary’ pericytes in the vast majority of the capillary bed, ‘transitional’ pericytes close to VSMCs and ‘stellate’ pericytes on post-capillary venules (Hartmann et al., 2020). Whether different pericyte subtypes have different functions, for example regulation of BBB permeability or control of CBF remains to be determined (Kisler et al., 2017).

Pericytes can constrict or relax, affecting capillary diameter, as discussed later in this review. Pericytes also promote vascular stability (Nishioku et al., 2009; Thomas and Augustin, 2009; Bell et al., 2010) and secrete basement membrane components (Virgintino et al., 2007). Studies have also underscored the importance of pericytes in modulating BBB integrity (Armulik et al., 2010; Daneman et al., 2010). Daneman et al. (2010) demonstrated that pericytes do not induce BBB-specific genes in ECs, but rather inhibit the expression of genes that promote vessel permeability. Pericytes have also been shown to affect functional aspects of the BBB, controlling both the structure of TJs and the rate of vesicular trafficking. Lack of pericytes (pericyte coverage between 20 and 40%) resulted in increased BBB permeability to water and a range of tracers of different molecular weights via increased endothelial transcytosis (Armulik et al., 2010). Similarly, a study using pericyte-specific Cre line crossed with mice carrying Cre-dependent human diphtheria toxin receptor showed that 40% pericyte coverage resulted in circulatory failure including BBB disruption, development of vasogenic edema and loss of CBF (Nikolakopoulou et al., 2019).

Following stroke, pericytes play a role in BBB remodeling and vessel stability (Su et al., 2019). Pericytes were shown to migrate away from brain microvessels in the first 2 h after occlusion of the internal carotid artery in cats (Gonul et al., 2002). Following photothrombotic occlusion of superficial cortical capillaries in mice, it was demonstrated that ischemia resulted in rapid activation of matrix metalloproteinase-9 (MMP-9) and plasma leakage at places where pericyte somata adjoined the capillary wall (Underly et al., 2017). The authors postulated that MMP-9 secreted from pericyte somata degraded underlying TJ complexes. This process was suggested as an intermediate step between leakage by transcytosis (transcellular leakage) and eventual TJ degradation (paracellular leakage). An important point raised by the authors, which would support findings from Gonul et al. (2002), is that pericytes may use MMP-9 to actively migrate from the endothelium to participate in revascularization (Underly et al., 2017). In addition, activation of PDGFR-β and Ang1/Tie2 signaling pathways are triggered by ischemic stroke, enhancing pericyte survival as well expression of TJ proteins in ECs, as reviewed elsewhere (ElAli et al., 2014). Finally, the control of endothelial transcytosis by pericytes following stroke requires further investigation. It has been proposed that pericytes may regulate transcytosis via expression of MFSD2A in brain ECs (Ben-Zvi et al., 2014; Keaney and Campbell, 2015; Sweeney et al., 2016; Chow and Gu, 2017). Importance of this cell–cell interaction in stroke remains to be comprehended, particularly in light of a recent study demonstrating the protective role of MFSD2A upregulation in rodent SAH (Zhao et al., 2020).

#### Effects of Stroke on Pericyte Function

The role of pericyte-dependent CBF regulation at the level of capillaries is currently debated, pericytes have the capacity to contract or relax, affecting capillary diameter in various physiological or pathological conditions (Hall et al., 2014; Hill et al., 2015; Cai et al., 2018). They possess the machinery necessary for cytoskeletal plasticity, including alpha-smooth muscle actin (α-SMA), tropomyosin and myosin. Pericytes are also sensitive to direct electrical stimulation or to neuronal activity via transmitters including NO, glutamate, noradrenalin, PGE2 or ATP (Peppiatt et al., 2006; Puro, 2007; Hall et al., 2014), and they respond by changes in intracellular Ca^2+^ by relaxation or constriction around the endothelium (Kawamura et al., 2003, 2004). A recent study reported that genetic ablation of pericytes in the mouse cerebral cortex correlated with 50% reductions in CBF responses to sensory stimulation (Kisler et al., 2020). A study by Hartmann et al. (2020) elegantly demonstrated, using two-photon live imaging, that optogenetic stimulation of pericytes decreased lumen diameter and CBF, but with slower kinetics than mural cells from upstream vascular beds.

The reactivity of pericytes is affected by stroke. Both physiological hypoxia and short-term hypoxia after stroke induce pericyte relaxation, a process modulated by PDGF-β, ATP, NO, and oxygen (Arimura et al., 2012; Cai et al., 2017). However, sustained hypoxic-ischemic damage leads to constriction and death of pericytes. Fernandez-Klett et al. (2013) reported that pericytes are rapidly lost 24 h after cerebral ischemia in both experimental (1-h tMCAo) and human stroke. *In vivo*, pericyte constriction/injury following ischemia-reperfusion was attributed to increased oxidative stress (Shojaee et al., 1999; Yemisci et al., 2009). OGD-induced ischemia in rat cerebellar slices triggered capillary constriction by pericytes followed by pericyte death, similarly 90 min of tMCAo in rats led to increased pericyte death in the lesioned hemisphere (Hall et al., 2014). Loss of pericytes also have profound effects on neurotrophic-dependent neuronal survival. This was demonstrated by genetic ablation of pericytes resulting in loss of pleiotrophin (PTN) expression; PTN is a pericyte-secreted growth factor and loss of this factor contributed to neuronal death in this study (Nikolakopoulou et al., 2019). Hence, pericytes can play a detrimental role in ischemia-reperfusion injury and thus represent a promising therapeutic target, as reviewed elsewhere (Cai et al., 2017; Su et al., 2019; Uemura et al., 2020).

### Effects of Stroke on Astrocytes

#### Effects of Stroke on Astrocyte Structure

Located between synapses and capillaries, astrocytes extend processes that physically link neighboring neurons with their surrounding blood vessels (Figure 1), allowing them to sense changes in the neuronal microenvironment and adjust the microvasculature accordingly (Attwell et al., 2010; Gordon et al., 2011; He et al., 2012). Several lines of evidence have implicated astrocytes in promoting and modulating the BBB identity of brain ECs (Abbott et al., 2006; Al Ahmad et al., 2011). In brief, perivascular astrocytes increase the tightness of TJs (Lee et al., 2003), promote the expression and localization of endothelial transporters (McAllister et al., 2001) and induce the expression of enzymes associated with the metabolic endothelial barrier (Abbott et al., 2006). Astrocytes are critical to neuronal survival and repair, a large part of this function being mediated through gap junction proteins that connect astrocyte networks into a cooperative functional syncytium (De Bock et al., 2017; Laird et al., 2017; Freitas-Andrade et al., 2019; Freitas-Andrade et al., 2020).

Generally, astrocytes are more resistant to hypoxic conditions than other CNS cells (Anderson and Nedergaard, 2003; Chen and Swanson, 2003). However, they are highly vulnerable to the coupling of acidosis and hypoxia during cerebral ischemia (Bondarenko and Chesler, 2001). In cell culture and *in vivo*, differences in sensitivity to hypoxia have been reported between different populations of astrocytes from different parts of the brain (Zhao and Flavin, 2000; Lukaszevicz et al., 2002; Shannon et al., 2007). Indeed, astrocytes differ between various regions of gray matter, or within a single brain region (Molofsky et al., 2012; Tsai et al., 2012; Clavreul et al., 2019; Batiuk et al., 2020). Astrocytes express gap junction proteins (Belliveau and Naus, 1994), neurotransmitter receptors, transporters (Zhou and Kimelberg, 2001; Matthias et al., 2003) and ion channels (Verkhratsky and Steinhauser, 2000). These specific molecular characteristics allow astrocytes to fulfill a range of homeostatic functions. However, this molecular diversity may bestow, to some astrocyte subtypes, vulnerabilities to stroke. One can also postulate that astrocytes are regulated by different cell types. For example, in a recent study, rats were subjected to global cerebral ischemia, performed by cardiac arrest of 10 min duration, then allowed to survive 2 years post-ischemia. After the 2 years, the authors found that in the hippocampal CA1 and CA3, and in the motor cortex, co-activation of both microglia and astrocytes was significant; however, in the resistant brain areas (that is, the dentate gyrus, sensory cortex, striatum, and dorso-lateral nucleus of the thalamus), significant activation was observed for astrocytes only (Radenovic et al., 2020). Similarly, in mice subjected to permanent MCAo, pericytes within the infarct area produced trophic factors activating astrocytes, thereby enhancing peri-infarct astrogliosis (Shibahara et al., 2020). This interplay between astrocyte and microglial and/or pericytes following ischemia remains elusive. Emerging technologies such as single-cell RNA sequencing, coupled with quantitative transcriptional genome-profiling, could molecularly define astrocytic subtypes and unmask mechanisms that affect astrocyte sensitivity to stroke.

In pathological conditions such as stroke, astrocyte survival has been correlated with neuronal survival (Chen and Swanson, 2003). Astrocytes secrete neurotrophic factors and, along with perivascular stromal cells, minimize damage to neighboring cells through formation of a glial scar (Krum et al., 2008; Fernandez-Klett et al., 2013). However, the glial scar can also be detrimental to functional recovery, by acting as a barrier to neuronal regeneration (Beck et al., 2008). Under ischemic conditions, astrocytes also secrete pro-angiogenic factors that promote the growth of new capillaries toward the infarcted tissue (Chow et al., 2001). Following brain injury, astrocytes upregulate glial fibrillary acidic protein (GFAP), an intermediate filament involved in astrocyte activation (Li et al., 2008). Interestingly, mice exposed to 1 hr of tMCAo coupled with a novel live imaging approach, Cordeau et al. (2008) reported that GFAP upregulation following ischemic brain injury may not have the same functional significance in male versus female mice (Cordeau et al., 2008). The authors showed that chronic estrogen deprivation (40 days after ovariectomy) resulted in a significant increase in GFAP upregulation in astrocytes after 24–72 h after reperfusion, compared with mice that were subjected to only 14 days of estrogen deprivation. However, the extent to which sexually dimorphic mechanisms affect astrocytic responses to stroke requires further investigation (Roy-O’Reilly and McCullough, 2018).

#### Effects of Stroke on Astrocyte Function

Astrocytes play important roles in homeostatic control of arterial blood pressure and CBF (Marina et al., 2020). Astrocytes are intimately associated with tens of thousands of synapses through highly ramified branches (Fields et al., 2015) and modulate CBF in response to synaptic activity (Anderson and Nedergaard, 2003). Astrocytes express metabotropic glutamate receptors (mGluRs) and sense glutamate release from synaptic clefts, and activation of mGluRs induces an increase in intracellular Ca^2+^ concentration spreading to the astrocytic endfeet (Zonta et al., 2003). These increases in Ca^2+^ concentration induce release of vasoactive factors from astrocytic endfeet and are dependent on the metabolic state of the neuronal microenvironment (Mulligan and MacVicar, 2004; Gordon et al., 2008).

Following stroke, profound functional changes occur at the level of astrocytes, which significantly affects neurovascular coupling. At the cellular level, post-stroke astrogliosis is noticeable around brain vessels (McConnell et al., 2019). At the molecular level, intracellular factors in astrocytes affect their ability to respond to neurometabolic needs. For instance, Howarth et al. (2017) demonstrated a novel mechanism of CBF regulation involving astrocytes and dependent on glutathione, a factor that is substantially reduced after stroke. When glutathione levels are reduced in conditions such as stroke, Ca^2+^-evoked release of PGE2 by astrocytic endfeet was decreased and vasodilation inhibited, an effect dependent of microsomal prostaglandin E synthase-1, downstream of COX-1 (Howarth et al., 2017).

A critical factor contributing to decreased CBF following stroke and implicating astrocytes are injury depolarizations, also known as Cortical Spreading Depressions or CSDs (Takano et al., 2007; Attwell et al., 2010). CSDs are slowly propagating waves of neuronal and glial depolarization (Lauritzen et al., 2011; Ayata and Lauritzen, 2015) that spontaneously occur within minutes after ischemic stroke and originate from the peri-infarct region (Dreier, 2011; Lauritzen et al., 2011; Kao et al., 2014; Lauritzen and Strong, 2016; Kirov et al., 2020). CSDs impair recovery in rodent stroke models (Risher et al., 2010; von Bornstadt et al., 2015) and correlate with clinical deterioration in stroke patients (Nakamura et al., 2010; Lauritzen and Strong, 2016). In the rat cerebral cortex, CSDs were shown to increase the vasoconstrictor 20-hydroxyeicosatetraenoic acid (20-HETE) which is generated in astrocytes from arachidonic acid, and known to induce constriction of VSMCs (Attwell et al., 2010; Fordsmann et al., 2013). It was postulated that 20-HETE secreted by astrocytes could have a significant impact on vascular function during stroke (Attwell et al., 2010). Astrocytic gap junctions have also been implicated in propagating CSDs and brain damage (Martinez and Saez, 2000; Rovegno and Saez, 2018).

Collectively, these studies show that cellular and molecular mechanisms normally associated with astrocytic regulation of CBF are hijacked following stroke. Dissection and understanding of these mechanisms represent another critical avenue for stroke research.

### Effects of Stroke on Microglia

Microglia play critical roles in both innate and adaptive immune responses in the CNS. They vigilantly monitor their microenvironment and perform homeostatic functions that are necessary for proper brain homeostasis (Nimmerjahn et al., 2005; Wake et al., 2009). Microglia are also involved in brain development, playing important roles in synaptic pruning, modulation of neurogenesis and myelination, as reviewed elsewhere (Tremblay et al., 2011; Wu et al., 2015; Hammond et al., 2018). A recent study using single cell transcriptomics discovered that mouse microglia are far more diverse than originally thought, comprising distinct subpopulations with unique molecular signatures (Hammond et al., 2019). While microglial ablation in the mature mouse brain does not affect BBB function (Parkhurst et al., 2013; Haruwaka et al., 2019), microglia can modulate BBB integrity in opposite ways during inflammation.

Following ischemic or hemorrhagic stroke, microglia dynamically transition into a reactive state (Eldahshan et al., 2019; Rawlinson et al., 2020). The initial leakage of blood serum components such as fibrinogen induces local activation of microglia. Microglia are finely tuned to sense any small disturbance in the BBB (Hines et al., 2009; Petersen et al., 2018), and their recruitment to blood vessels occurs within 6 h of reperfusion with significant accumulation in perilesional tissue. After 24 h of reperfusion, microglia fully enwrap small blood vessels in the peri-infarct region (Jolivel et al., 2015). Individual perivascular microglia displayed intracellular vesicles containing CD31-positive inclusions, suggesting phagocytosis of brain ECs, which was correlated with BBB breakdown as shown by the extravasation of Evans blue from perfused vessels. At 72 h post-MCAo, blood vessel degradation was complete and remaining vascular debris were cleared by microglia and invading immune cells (Jolivel et al., 2015). Following stroke, reactive microglia also secrete MMP-9 and MMP-3, proteases that can break down the basement membrane surrounding brain–blood vessels and exacerbate BBB leakage (Yenari et al., 2010), as discussed below.

Following ICH, blood invading the brain parenchyma induces a rapid inflammatory response from microglia. Activated microglia develop into an M1-like phenotype resulting in production of pro-inflammatory cytokines such as [interleukin (IL)-1β, IL-6, IL-12, IL-23, tumor necrosis factor alpha (TNF-α)], chemokines, redox molecules (NADPH oxidase, phagocyte oxidase, inducible NO synthase), costimulatory proteins (CD40), and major histocompatibility complex II (MHC-II) (Zhang et al., 2017). In the acute phase of ICH, both in the clinical and experimental rodent models, proinflammatory factors are present in the brain starting 3 h after ICH and peaking at 3 days. Due to their proinflammatory phenotype, M1 microglia are linked to short-term brain damage. Within 1 week, a M1-to-M2 microglial phenotypic switch occurs (Lan et al., 2017). M2-like microglia are associated with anti-inflammatory and phagocytic functions and assist in the clearance of the haematoma. Microglia can also be activated by IL4/IL3 to the M2 polarization state, which produces anti-inflammatory mediators IL-10, transforming growth factor beta (TGFβ), and glucocorticoids (Zhang et al., 2017). Several factors have been implicated in inducing microglial polarization including, nuclear factor-κB (NF-κB), signal transducer and activator of transcription (STAT1–STAT6), high mobility group protein B1 (HMGB1) as well as PGE2 (Lan et al., 2017). Finally, studies have shown that age, environmental factors and sex differences can influence microglial responses and polarization to injury (Crain et al., 2013; Bisht et al., 2016; Lan et al., 2017). Taken together, this shows that various conditions may have a profound impact on the responsiveness of microglia following stroke.

### Effects of Stroke on Perivascular Macrophages

Although different from microglia, the function of brain perivascular macrophages (PVMs) are of growing interest in stroke research. PVMs are myeloid cells located in the perivascular space surrounding cerebral blood vessels (Faraco et al., 2017). In the healthy brain, PVMs contribute to BBB integrity and help regulate infiltration of large molecules into the brain through scavenger activity (Mendes-Jorge et al., 2009). PVMs have largely been implicated in their role as scavengers in the context of Alzheimer’s disease and CNS infection, however, there is increasing evidence for their role in the regulation of CBF, vascular function and stroke pathogenesis. Depletion of PVM has been shown to prevent changes in vascular structure associated with chronic hypertension (Pires et al., 2013). Additionally, PVMs were shown to promote BBB degradation through ROS production in a mouse model of hypertension, which could be reversed by depleting PVMs, effectively reducing oxidative stress, improving CBF dysfunction, restoring neurovascular coupling, and rescuing cognitive impairment (Faraco et al., 2016). In post-mortem tissues, cells positive for the PVM marker CD163 were found accumulated in brains with ischemic, but not hemorrhagic, lesions (Holfelder et al., 2011). Furthermore, CD163-positive cells isolated from rats following 1-h tMCAo followed by 16-h reperfusion showed upregulation of the HIF-1 pathway, as well as of genes encoding the ECM and leukocyte chemoattractants (Pedragosa et al., 2018). Depletion of PVMs reduced granulocyte infiltration, BBB permeability and VEGF expression (Pedragosa et al., 2018). Because VEGF promotes migration of cells to participate in angiogenesis, it is possible upregulation of HIF-1 and VEGF by PVMs is pathological in the acute phase following ischemic stroke. It has been hypothesized that activation of PVMs in cerebrovascular pathologies may initially be protective through their phagocytic activity, but may in turn be detrimental with repeated long-term activation (Koizumi et al., 2019). Further research is required to fully elucidate the role of PVMs in the context of stroke.

### Effects of Stroke on the Basement Membrane

The basement membrane forms a three-dimensional protein network composed of laminins, collagen, nidogen and heparan sulfate proteoglycans (HSPGs) that mutually support interactions between ECs, pericytes and astrocytes (Figure 1) (Thomsen et al., 2017). The basement membrane functions as a second barrier, limiting movement between the blood and the brain. At the NVU, ECs, astrocytes and pericytes synthesize and deposit different laminin isoforms in the basement membrane, which have been shown to modulate BBB function (Gautam et al., 2016, 2019). Penetrating arteries and parenchymal arterioles are surrounded by a basement membrane composed of two distinct entities: the basement membrane produced by the endothelium, and the parenchymal membrane located between vascular smooth muscle cells (VSMCs) and astrocytes, produced by pial cells and astrocytic endfeet. Pericytes also contribute to basement membrane formation by producing and secreting ECM proteins (Yao, 2019).

Several lines of evidence suggest that integrin matrix adhesion receptors expressed by ECs and astrocytes exhibit dynamic cellular influences (Milner et al., 2008; McCarty, 2020). In addition, matrix adhesion by endothelial β1-integrin receptors affect claudin-5 expression and regulate BBB permeability (Osada et al., 2011). Interestingly, studies have also indicated the importance of the basement membrane in cerebrospinal fluid regulation (Morris et al., 2016; Albargothy et al., 2018; Howe et al., 2019). Impaired basement membrane integrity is a significant contributor to neuronal loss after stroke.

The ECM of the basement membrane plays a role in limiting the transmigration of erythrocytes during hemorrhage, and of leukocytes during inflammation. Following ischemic stroke, MMPs produced by activated ECs and pericytes degrade the basement membrane (Thomsen et al., 2017; Kang and Yao, 2020). Other proteinases, including plasminogen activators, heparinases and cathepsins also contribute to ECM degradation. The proteolytic breakdown of ECM proteins such as laminin-5 or type IV collagen exposes cryptic epitopes that promote EC and pericyte migration (Hangai et al., 2002). A recent study highlighted the complex molecular cascades and plethora of genes induced by stroke that are in relation to ECM and NVU integrity (Aleithe et al., 2019). Aging is also an important factor in basement membrane integrity after stroke. TGF-β signaling in hypoxic astrocytes induces basement membrane fibrosis and chronically impairs perivascular CSF distribution, specifically in aged animals after permanent MCAo (Howe et al., 2019), providing a new mechanism by which brain injury can lead to prolonged functional impairment in the elderly.

Interestingly, disruption of astrocyte-derived laminin expression resulted in spontaneous hemorrhagic stroke in deep brain regions (basal ganglia), which are similarly affected in human patients. Chen et al. (2013) generated conditional knockout mice in which astrocytes do not express laminin γ1 chain, an essential subunit of most laminins (Durbeej, 2010). Lack of astrocyte-derived laminin γ1 resulted in impaired VSMC differentiation and decreased levels of contractile proteins in VSMCs around small arteries and arterioles (diameter 8–20 μm), but only in the striatum. The authors observed that while mutant astrocytes throughout the brain did not produce laminin, hemorrhaging occurred only in the basal ganglia. In the normal brain, penetrating arteries and arterioles are surrounded by a basement membrane composed of two distinct entities: the basement membrane produced by the endothelium and the parenchymal membrane. As arteries branch into small arteries, and small arteries ramify into arterioles, the contribution of the pia meninges decrease. At the capillary level, there are no pia meninges, and the basement membrane between the astrocytic endfeet and VSMC become very thin, at some points along the capillary endfeet directly contact VSMCs or ECs (Yao, 2019). It was postulated that, due to the close relationship between astrocytes and VSMCs in the striatal vasculature, the lack of astrocyte-derived laminins had a direct effect on the underlying VSMCs within this brain region (Chen et al., 2013). In contrast, this close relationship between astrocytes and VSMCs was not observed in the cerebral cortex. The phenotype presented by the transgenic animals appears similar to abnormalities found in human hypertensive hemorrhagic patients in the striatum (Chen et al., 2013). More recently, Gautam et al. (2020) demonstrated in mutant mice lacking mural cell-derived laminin that the latter attenuates BBB damage in ICH via decreasing caveolin-1 and transcytosis.

Following 6 h of tMCAo, basement membrane degradation was observed 10 min after reperfusion, and basement membrane loss was detected as early as 1–3 h after ischemia (Yao, 2019). In a non-human primate study after middle cerebral artery occlusion/reperfusion both MMP-2 and -9 are significantly upregulated and digest ECM proteins of the basement membrane, affecting BBB integrity (Heo et al., 1999). A possible harmful consequence of MMP-9 activation during acute stroke treatment is that rtPA can leak out of the vessel through the permeable BBB and substantially further enhance MMP-9 levels, resulting in hemorrhage (Tsuji et al., 2005; Yao, 2019).

Cathepsin B and L proteases are enhanced soon after stroke onset and degrade heparan sulfate proteoglycans (HSPGs) (Becker et al., 2015). Reduction of HSPG has a dramatic effect on the BBB, as the HSPG Agrin is known to stabilize adherens junctions in mouse brain ECs (Steiner et al., 2014). While proteases activated during stroke may have detrimental effects during initial stages, they also play an important role in angiogenesis and vascular remodeling (Thomsen et al., 2017). MMPs are integral players in angiogenesis, breaking down ECM proteins to facilitate endothelial tip cell and pericyte migration. It has also been demonstrated that degraded fragments of the HSPG Perlecan reduce neuronal death and infarct volume, as well as enhance angiogenesis (Lee et al., 2011; Bix et al., 2013).

Targeting MMPs has some potential therapeutic benefits (Chaturvedi and Kaczmarek, 2014). Minocycline is a lipophilic tetracycline and was shown to inhibit MMP-9 activity and expression in rats subjected to 3 h of tMCAo (Machado et al., 2006). In this study, minocycline was administered after the stroke and given at a clinically relevant concentration (intra-peritoneal minocycline 45 mg/kg). Although, the authors did not show whether minocycline reduced infarct damage, minocycline later appeared neuroprotective in several models of brain injury (Naderi et al., 2020) with demonstrated efficacy in acute stroke patients (Malhotra et al., 2018). Moreover, as mentioned previously, MMP-9 has been associated with hemorrhagic transformation in the setting of tPA therapy (Aoki et al., 2002). MMP-9 is associated with BBB breakdown and subsequent vasogenic edema, and an MMP-9 polymorphism was shown to confer susceptibility to ischemic stroke in a Chinese population (Jiang et al., 2020). HIBISCUS-STROKE is a cohort study including acute ischemic stroke patients with large vessel occlusion treated with mechanical thrombectomy following admission magnetic resonance imaging (MRI) (Mechtouff et al., 2020). In this study, MMP-9 levels were assessed to determine whether it correlated with infarct growth and hemorrhagic transformation. The study showed that MMP-9 levels measured 6 h after admission predicted infarct growth and hemorrhagic transformation (Mechtouff et al., 2020).

In summary, sudden and sustained interruption of blood flow to the brain induces dynamic highly complex cellular and molecular responses in the NVU (Figure 1C and Table 1). While the disruption at the NVU is catastrophic, the mechanisms triggered by ischemia or hemorrhage are set in motion in order to restore homeostatic balance. Increased BBB permeability and basement membrane breakdown due to secretion of MMPs by ECs, pericytes and astrocytes facilitate cell migration and vascular remodeling. Fibrinogen and other blood components leaking into the parenchyma activates microglia and promote phagocytosis of cellular debris. Secreted factors by these cells as well as components of the basement membrane induces angiogenesis and capillary network formation after stroke.

**TABLE 1:** Major features (non-exhaustive list) of structural and functional remodeling of the neurovascular unit following stroke.

		Selected references
**Structural NVU Remodeling**		
Ischemic Stroke	– Reparative angiogenesis primarily in the peri-infarct. – Biphasic BBB breakdown: (1) Increased caveolae-mediated transcytosis. (2) Tight junction breakdown. – Secretion of MMPs by pericytes, ECs, and microglia promotes degradation of the basement membrane and TJ disruption, leading, to increased BBB permeability and edema. – Secreted MMPs also facilitate angiogenesis and vascular remodeling by promoting EC and pericyte migration. – Basement membrane fibrosis induced by TGF-β. – Astrocytes contribute to glial scar formation which is both beneficial and detrimental to nearby cells. – Astrocytes upregulate GFAP soon after stroke and secrete neurotrophic and proangiogenic factors. – Pericytes secrete trophic factors that contribute to astrogliosis. – Leakage of blood-borne factors into brain parenchyma results in rapid microglia activation that enwrap and phagocytose ECs in the peri-infarct region.	Chow et al., 2001; Hangai et al., 2002; Beck et al., 2008; Krum et al., 2008; Yu et al., 2010; Yenari et al., 2010; Jiao et al., 2011; Ben-Zvi et al., 2014; ElAli et al., 2014; Knowland et al., 2014; Jolivel et al., 2015; Choi et al., 2016; Nahirney et al., 2016; Thomsen et al., 2017; Underly et al., 2017; Eldahshan et al., 2019; Howe et al., 2019; Munji et al., 2019; Yao, 2019; Shibahara et al., 2020.
Hemorrhagic stroke	– ECs proliferate around hematoma following ICH. – BBB breakdown and tight junction disruption. – Blood in parenchyma results in rapid microglia activation to a pro-inflammatory phenotype, which eventually polarize to an anti-inflammatory phenotype. – Mutations in genes that encode basement membrane proteins are associated with ICH. – Loss of astrocyte-derived basement membrane proteins is associated with hemorrhagic stroke in deep brain regions. – MMP-9 implicated in hemorrhagic transformation following treatment for ischemic stroke. – VEGF can also increase BBB permeability, which may help peripheral macrophages infiltrate into the brain.	Manoonkitiwongsa et al., 2001; Gould et al., 2006; Chen et al., 2013; Fu et al., 2014; Lan et al., 2017; Zhang et al., 2017; Gautam et al., 2020; Mechtouff et al., 2020.
**Functional NVU Remodeling**		
Ischemic stroke	– Acute loss of CBF initiates vascular remodeling via eNOS. – Acute hypoxia induces pericyte relaxation, however, sustained hypoxia leads to pericyte constriction and death. – Functional changes in astrocytes significantly affect NVC. – Decrease in glutathione impairs astrocytic regulation of CBF. – Astrocytes implicated in propagating CSD and VSMC constriction contributing to decreased CBF. – Cell death of perivascular neurons exacerbates brain damage and leads to neurovascular uncoupling. – Hypoxia activates and stabilizes HIFs, upregulating VEGF signaling and promoting angiogenesis. – Angiogenic response provides a scaffold for neuronal regeneration, mediated by neural precursor cells.	Marti et al., 2000; Attwell et al., 2010; Arimura et al., 2012; Fernandez-Klett et al., 2013; Hall et al., 2014; O’Donnell, 2014; Hoffmann et al., 2015; Reeson et al., 2015; Howarth et al., 2017; Cai et al., 2018; Rovegno and Saez, 2018; McConnell et al., 2019; Tornabene et al., 2019.
Hemorrhagic stroke	– VEGF and its receptors upregulated persistently. – Increased VEGF increases vessel density and improves stroke outcome. – Beneficial effects of VEGF mediated through aquaporin-4. – Morphology of newly formed vessels resemble that of the developing brain.	Josko, 2003; Tang et al., 2007; Chu et al., 2013; Sugimoto and Chung, 2020.

**Selected references are displayed. BBB, blood–brain barrier; TJ: tight junction; MMPs, matrix metalloproteinases; EC, endothelial cell; ICH, intracerebral hemorrhage; NVC, neurovascular coupling; NVU, neurovascular unit; CBF, cerebral blood flow; CSD, cortical spreading depression; VSMC, vascular smooth muscle cell; HIF, hypoxia-inducible transcription factors; VEGF, vascular endothelial growth factor*.*

### Regulation of Angiogenesis Following Stroke

#### Lessons From Developmental Biology

To gain further insight into angiogenesis in the injured/ischemic adult brain, it is critical to understand developmental angiogenesis, given that developmental processes are re-activated following stroke (Lee et al., 2004; Gonzenbach and Schwab, 2008; Milner et al., 2008).

Stroke triggers a complex set of cellular and molecular responses that evolve from minutes to days. Energy supply and ionic balance are immediately compromised in the ischemic core, leading to rapid neuronal demise. Directly surrounding the infarct core, the peri-infarct region (also referred to as “ischemic penumbra”) is a territory that still receives limited perfusion by collateral blood vessels. Due to the inadequate blood supply, this peri-infarct region is functionally silent, yet potentially salvageable (del Zoppo et al., 2011). In the early 1990’s, a post-mortem study on human brains demonstrated that stroke activates angiogenesis mostly in the peri-infarct region, and a higher blood vessel count correlated with longer survival time (Krupinski et al., 1994). Subsequent human studies demonstrated a correlation between improved stroke outcome and levels of circulating pro-angiogenic factors (Lee et al., 2010; Navarro-Sobrino et al., 2011).

During early development, brain vascularization is mediated through ingression of blood vessels in the presumptive cerebral cortex from a superficial vascular plexus, with hypoxia and genetic programs as driving forces. Blood vessels within the brain then sprout and expand into vast highly connected networks and remodel into a complex vascular tree characterized by an arterial and venous hierarchy (Carmeliet and Tessier-Lavigne, 2005; Tata et al., 2015). As brain tissue expands and oxygen diffusion from neighboring capillaries is insufficient, a mild hypoxia promotes activation of hypoxia-inducible transcription factors (HIFs). HIFs are heterodimeric proteins consisting of a constitutive subunit HIF-1β as well as either a HIF-1α or HIF-2α subunit. HIF-1α and -2α subunits are rapidly degraded in normoxia, which is initiated by the hydroxylation of two conserved prolyl residues in the HIF-α subunits (Tomita et al., 2003). When cellular oxygen concentration is reduced, HIF-1α and -2α protein levels increase dramatically. More than 1,000 genes are directly transactivated by HIFs in response to hypoxia (Semenza, 2014; Rattner et al., 2019). HIFs induce the expression of angiogenic genes that act both on the nascent cerebrovascular system, as well as developing neurons. The intimate relationship between the vasculature and neurons is established early during development. For example, signaling factors associated with axonal guidance (Netrins, Semaphorins, and Ephrins) as well as angiogenic factors (VEGFs) are common signals orchestrating the regulation of both vessels and neuronal development (Gu et al., 2005; Oh and Gu, 2013). Detailed reviews about neuro-vascular development can be consulted (Tam and Watts, 2010; Eichmann and Thomas, 2013; Andreone et al., 2015; He et al., 2018; Paredes et al., 2018; Coelho-Santos and Shih, 2020).

#### Angiogenesis After Ischemic Stroke

Similar to the developing brain, low O_2_ levels increase the stability and activity of HIFs in vulnerable cells of the peri-infarct region, triggering angiogenesis from non-affected tissue and pial vessels. New vessels grow through the hypoxic micro-environment of the penumbra into the core of the infarct (Marti et al., 2000). Post-stroke HIF activation induces the expression of several angiogenic and inflammatory factors including VEGF. Serum VEGF is significantly increased in ischemic stroke patients (Dassan et al., 2012; Paczkowska et al., 2013), in whom highest VEGF expression occurs 7 days post-stroke, and remains significantly elevated 14 days after stroke (Slevin et al., 2000; Matsuo et al., 2013). VEGF and its receptors (VEGFR-1 and -2) play a central role in initiating CNS angiogenesis, stimulating endothelial cell survival, proliferation and migration. In permanent MCAo mouse model, VEGF expression was detected within the first 24 h after occlusion in hypoxic peri-infarct tissues and in the pia above the infarcted area. Within the same brain regions, VEGFR-1 and subsequently VEGFR-2 were increased 48 h after MCAo (Marti et al., 2000). After 48 and 72 h of ischemia, a dramatic increase in proliferating ECs was measured within the peri-infarct area as well as the pial surface. The authors reported that VEGFRs were induced mainly in ECs, but that VEGFR-2 was also detected in hippocampal neurons in both the ipsilateral and contralateral hemispheres, suggesting that the VEGF/VEGFR pathway could be associated with neuroprotection. Other studies using either permanent or transient MCAo showed similar spatio-temporal dynamics in VEGF/VEGFR expression (Plate et al., 1999; Beck et al., 2002). Taken together, these studies indicate that ischemia is a significant driving force of angiogenesis during the initial stages of stroke and is mediated by VEGF and its receptors.

While VEGFR-1 is involved in attenuating the effects of VEGF (Kearney et al., 2002; Meyer et al., 2006) and modulating inflammatory responses (Cardenas-Rivera et al., 2019), VEGFR-2 activation, induces intracellular pathways associated with EC activation and neuroprotection. VEGFR-2-PI3K-Akt signaling pathway was linked to neuronal survival and reduced infarct size in mice subjected to 90 min of tMCAo (Kilic et al., 2006). However, it was also shown that VEGFR-2 mediated PI3K-Akt signaling induced BBB permeability (Kilic et al., 2006). While the benefits of VEGF-dependent activation of VEGFR-2 have been demonstrated, the detrimental effects on vascular permeability are also well known (Zhang et al., 2002; Reeson et al., 2015; Geiseler and Morland, 2018). Due to these contrasting effects, the use of VEGF as a therapeutic strategy in stroke has been challenging.

In addition, a role for ADAMTS13 in reparative angiogenesis after ischemic stroke was recently discovered *in vivo*. Normally after vascular injury, von Willebrand factor is secreted as hyperactive ultralarge multimers that are rapidly cleaved by ADAMTS13 into less reactive fragments (Crawley et al., 2011). Following permanent MCAo, *Adamts13*^–/–^ mice displayed reduced neovascularization, reduced brain capillary perfusion, as well as accelerated BBB breakdown (Xu et al., 2017).

#### Angiogenesis After Hemorrhagic Stroke

The two types of hemorrhagic stroke are: intracerebral hemorrhage (ICH), defined as bleeding into the brain parenchyma, and subarachnoid hemorrhage (SAH) caused by bleeding into the cerebrospinal fluid (CSF)-containing sulci, fissures and cisterns (Smith and Eskey, 2011). There are marked differences in neurological cascade of events between ischemic and hemorrhagic strokes (Qureshi et al., 2009). However, both hemorrhagic and ischemic strokes share common angiogenic mechanisms. Tang et al. (2007) demonstrated that angiogenesis in rat brains subjected to collagenase-induced ICH was similar to those observed following ischemic stroke. Seven days after collagenase injection into the right globus pallidus, enlarged and thin-walled microvessels appeared along the border of the hematoma and continued to grow into the core, and then spread all over the clot by 21 days. Endothelial cell proliferation was also observed around the hematoma 2 days after collagenase injection and peaked from 7 to 14 days. Within the same time frame, VEGF as well as VEGFR-1 and -2 mRNA were detected as early as 2 days after ICH; mRNA levels peaked at 21 days and persisted for at least 28 days post-ICH (Tang et al., 2007). Interestingly, the authors noted that newly formed microvessels displayed an enlarged and thin-walled morphology, reminiscent of those found in the developing brain. Similarly, angiogenesis was observed in rats subjected to a SAH stroke paradigm, and expression of VEGF was induced by hypoxia resulting from vasospasm (Josko, 2003). Similar to ischemic stroke, CSD also occurs in hemorrhagic stroke (Sugimoto and Chung, 2020). Subsequent ICH studies suggested that angiogenesis may have therapeutic benefits (Lei et al., 2013; Pan et al., 2018). For instance, treatment with EGb761, a Ginkgo biloba extract, increased microvessel density and promoted neuroprotection in mice subjected to ICH induced by collagenase injection (Pan et al., 2018). EGb761 treatment enhanced VEGF expression, while inhibition of this VEGF expression negatively affected stroke outcome (Pan et al., 2018). Similarly, the effects of VEGF inhibition on collagenase-induced ICH in rats was demonstrated through pharmacological inhibition of high-mobility group box 1 protein (HMGB1), a member of the damage-associated-molecular-pattern (DAMP) family of proteins. Inhibition of HMGB1 resulted in reduced levels of VEGF and nerve growth factor (NGF), and reduced recovery of neurological function following ICH (Lei et al., 2013). Beneficial effects of VEGF on brain edema following ICH were also reported (Chu et al., 2013). In this particular study, ICH was induced by microinjecting autologous whole blood into the right striatum of transgenic aquaporin-4 (AQP4) Wild-Type (AQP4^+/+^) and knockout (AQP4^–/–^) mice. One day after injury, recombinant human VEGF injected intracerebroventricularly induced AQP4 expression in the striatum of AQP4^+/+^ mice 1 day after VEGF injection, and peaked at 3 days. AQP4 was still present 7 days post-injection and concentrated in glial endfeet surrounding the hematoma (Chu et al., 2013). While AQP4^+/+^ mice injected with VEGF showed reduced neurological deficits and decreased brain edema following ICH at 1, 3, and 7 days post-treatment, AQP4^–/–^ ICH mice did not benefit from VEGF injection. Moreover, this study demonstrated that VEGF did not affect BBB permeability after ICH. In view of these studies, VEGF may have therapeutic potential for ICH.

#### Reparative Angiogenesis as Support for Post-stroke Neurogenesis

A key role for angiogenic responses to ischemic injury is to provide a scaffold for neuronal regeneration. Proper cell–cell communication within vascular niches of neurogenesis is crucial for regenerative mechanisms in the adult brain. Close reciprocal relationships between brain ECs and neural progenitor cells (NPCs) regulate neurogenesis in both the developing and adult brain (Goldman and Chen, 2011; Licht and Keshet, 2015; Segarra et al., 2015, 2018; Tata and Ruhrberg, 2018). NPCs secrete proangiogenic factors that promote brain vascularization, and brain ECs instruct NPCs to proliferate, differentiate, or remain quiescent through release of angiocrine messengers including NO, BDNF, stromal-derived factor 1, or angiopoietin 1 (Ohab et al., 2006; Goldman and Chen, 2011). Stroke triggers a regenerative response in the peri-infarct region, adjacent to the core area of cell death. A focal cortical stroke in mice induced a strong neurogenic response with induction of GFAP-expressing NPCs in the subventricular zone, followed by migration of neuroblasts along existing and newly formed vascular beds toward the peri-infarct cortex (Ohab et al., 2006; Ohab and Carmichael, 2008). Following this important discovery that angiogenesis and neurogenesis are causally linked in the post-stroke niche, several studies have investigated these complex structural and molecular neuro-vascular interactions, as recently reviewed elsewhere (Fujioka et al., 2019; Hatakeyama et al., 2020). Overall, this supports the idea that enhancing post-stroke angiogenesis might represent a valuable strategy to promote post-stroke functional recovery.

In summary, angiogenesis is a multistep process involving basement membrane breakdown, cell proliferation and migration, capillary morphogenesis, vascular maturation and vascular pruning and cellular apoptosis. Similar angiogenic mechanisms are triggered in both ischemic and hemorrhagic brain injury. Many of these mechanisms are also critical during brain development and are similarly induced by ischemia. Importantly, formation of new capillaries, through angiogenic processes, provide a scaffold for neuronal stem cell recruitment both during brain injury and CNS development.

## Sex Differences in Cerebrovascular Outcomes of Stroke

Sex differences in brain morphology, function and disease are eliciting growing interest, but very little is known about the cellular and molecular underpinnings of sex differences in vascular outcomes of stroke. Biological sex markedly influences CBF as well as the prevalence and progression of cardiovascular diseases, including stroke (Krause et al., 2006; Cosgrove et al., 2007; Hofer et al., 2007; Cowan et al., 2017). It is well recognized that stroke differentially affects women and men. Although men have a higher incidence of stroke compared to age-matched pre-menopausal women, epidemiological studies show that most women have strokes when they are post-menopausal, resulting in increased stroke severity, worse psychological outcomes, and higher rates of disability (Persky et al., 2010; Turtzo and McCullough, 2010; Barker-Collo et al., 2015; Ahnstedt et al., 2016; Madsen et al., 2019; Wang et al., 2019). Despite this, the effects of sex hormones on cerebrovascular regulation in the healthy and ischemic brain have yet to be fully comprehended.

The concept of sex differences in neuro-vascular research was not well appreciated until recently. A common finding is an increased baseline CBF in women versus men (Cosgrove et al., 2007; Ghisleni et al., 2015). Women also display greater perfusion during cognitive tasks (Gur et al., 1982; Esposito et al., 1996), and better autoregulation of CBF as they age (Deegan et al., 2011). Yet, the underlying causes of these sex differences are unknown. Sex differences in CBF are due in part to the combined modulation by steroid hormones. Estradiol, testosterone and dehydroepiandrosterone sulfate are modulators of brain perfusion (Ghisleni et al., 2015). Testosterone mainly exerts vasoconstrictive effects, and its supplementation decreases CBF in post-menopausal women. 17β-estradiol (E2) is the most abundant and potent estrogen in mammals. Binding of E2 to its receptor ERα increases NO production through upregulation of eNOS (Miyazaki-Akita et al., 2007), as well as via decreasing the concentration of NO-scavenging superoxide anion (Novella et al., 2012). eNOS is modulated by ERα activation via: (1) typical ERα signaling with nuclear translocation of intracellular receptors, leading to increased eNOS gene (*Nos3*) expression, or (2) the lesser-studied stimulation of membrane-bound ERα leading to phosphatidylinositol-3-kinase pathway stimulation and eNOS activation (Novella et al., 2012). Signaling through these pathways results in increased bioavailability of NO, a potent relaxant of VSMCs and therefore vasodilator (Chen et al., 2008; Moncada and Higgs, 1993).

Lower incidence rates of stroke in pre-menopausal women has been linked to a protective effect of estrogens (Turtzo and McCullough, 2010), and after menopause rates of stroke dramatically increase (Lisabeth and Bushnell, 2012; Xu J. et al., 2016). As women have a longer life expectancy, they account for 60% of stroke events when incidence rates are adjusted for age (Reeves et al., 2008). Following menopause, estrogen production by the ovaries decreases by >50%. This has supported the theory that estrogens are protective in CVD, which has been attributed in part to the ability of estrogens to enhance NO production via stimulation of eNOS (Krause et al., 2006; Nevzati et al., 2015).

Protective roles of estrogens have been reported in a variety of animal models of cerebral ischemia. Numerous studies show that estrogen treatment or activation of estrogen receptors reduces lesion size in these animal models (Yang et al., 2000; McCullough et al., 2001; Selvaraj et al., 2018; Xiao et al., 2018) while removing endogenous estrogen through ovariectomy (Ovx) worsens their outcomes (Alkayed et al., 1998; Fukuda et al., 2000). Furthermore, female rats that undergo tMCAo during the proestrus phase of their estrous cycle (i.e., highest estradiol levels) have smaller infarcts than females in other phases of the cycle (Liao et al., 2001). Estrogen supplementation of Ovx rodents prior to stroke has also been found to preserve BBB integrity by reducing EC death and preventing the loss of TJ proteins (Liu et al., 2005; Shin et al., 2016). *In vitro*, estradiol protects the endothelium by reducing mitochondrial reactive oxygen species (ROS) production following ischemic injury (Razmara et al., 2008; Guo et al., 2010). These protective mechanisms may contribute to preserving not only neuronal health, but also vascular health, during and following cerebral ischemia.

Overall, there are very few mechanistic investigations on disparities between sexes in post-stroke CBF outcome. Ovx rats displayed significantly lower CBF following tMCAo compared to intact females. Upon estrogen supplementation, CBF in Ovx rats could be rescued 1 day post-stroke (Yang et al., 2000). Long-term estrogen treatment increases eNOS expression in cerebral blood vessels from male and female rats (McNeill et al., 1999), suggesting that NO may play a protective role through vasorelaxation. In contrast, males treated with estrogen immediately following tMCAo had increased CBF up to 10 min following stroke, but not past 90 min (McCullough et al., 2001), but not past 90 min, suggesting that modulation of hormones might not be a viable therapeutic option. Additionally, following photothrombotic distal MCAo, female rats showed quicker vascular remodeling of occluded and peripheral vessels compared to males (Yang et al., 2019). Only one study has shown that CBF values of females are higher following stroke compared to males and Ovx females, and the mechanism behind this difference has yet to be elucidated (Alkayed et al., 1998).

Despite the promising effects of estrogens in rodent stroke models, hormone therapy containing either combined estrogen and progesterone, or estrogen alone, increases the risk of ischemic stroke by 40–50% in healthy postmenopausal women (Wassertheil-Smoller et al., 2003; Hendrix et al., 2006; Hale and Shufelt, 2015). In this case, the stroke is most often thrombotic, which is attributed to decreased plasma levels of endogenous circulating anticoagulants in response to high estrogen levels (Mendelsohn and Karas, 1999). There is also the timing hypothesis for hormone therapy, which suggests that treatment with exogenous estrogens and progesterone causes more harm when EC viability is already compromised, as is often the case in aging women (Lisabeth and Bushnell, 2012). Additionally, hormone replacement therapy using estrogens can increase the risk of ovarian and breast cancer (Brown et al., 2018). For these reasons, hormone replacement therapy to reduce stroke risk in post-menopausal women is not recommended. Therefore, it is critical to better understand how sex hormones regulate vascular function in order to refine future therapies. Switching to novel targets might represent safer options, but further preclinical research is warranted. Known eNOS enhancers (e.g., AVE3085 and AVE9488) that have been beneficial for peripheral cardiovascular disease (CVD) in animal studies might prove particularly efficient in post-menopausal women.

In summary, although existing literature on sex differences in stroke severity and mortality are somewhat contradictory, women suffer from worse functional outcomes and have high levels of long-term disability. Animal models do not entirely reflect what is observed in the clinic and estrogen therapy, while beneficial in rodent experiments, failed to translate into the clinical setting. Many factors may influence sex-specific responses to stroke including epigenetics, immune responsiveness, inflammation and chromosomal contributions. This area of research has been largely overlooked, and given the significant impact stroke has in women it is imperative that more research is conducted.

## Concluding Remarks

### Limitations of Preclinical Stroke Research

The majority of preclinical work on cerebrovascular stroke outcomes has been performed in anesthetized healthy rodents, often using solely males. Moreover, two important limitations of preclinical studies on sex differences in stroke have been (i) the use of young animals and (ii) the misconception that Ovx (i.e., model of reduced steroid influence) mimics human menopause. Aging is a key risk factor for stroke, together with several comorbidities such as hypertension and atherosclerosis that develop with age. The use of young healthy male rodent models, not reflective of the human condition, is a contributing factor to the failure to translate drugs into the clinic. While these concerns are addressable by using rodent cohorts that better mimic the human population most often affected by stroke, there are inherent problems that must be accounted for in preclinical stroke models.

Experimental MCAo is the most commonly used animal model of ischemic stroke, which consists of either permanent (without reperfusion) or transient (with reperfusion) occlusion of the middle cerebral artery (MCA). While reproducible, MCAo has important translational limitations. As typically used, MCAo creates large infarcts equivalent to malignant human brain infarction (Carmichael, 2005). Furthermore, permanent and complete occlusion of the MCA does not accurately represent human ischemic stroke, and the transient model that allows for quick reperfusion is more representative of global ischemia conditions rather than a focal ischemic stroke (Sommer, 2017). While MCAo has a similar inflammatory profile as seen in humans and is useful to assess neuroprotection, as it allows for sensitive measures of neuronal death, it is not recommended for stroke recovery studies that rely on behavioral outcomes (Corbett et al., 2017; McCabe et al., 2018). However, it has recently been suggested that the MCAo model may be useful for mimicking the conditions associated with endovascular treatment of ischemic stroke (Sommer, 2017).

Accordingly, it is preferable to create focal ischemia using the photothrombotic (PT) or endothelin-1 (ET-1) stroke models, which are both highly recommended by recent international consensus panels (Tennant and Jones, 2009; Roome et al., 2014; Corbett et al., 2017). Stereotaxic injection of the peptide ET-1, a potent vasoconstrictor, restricts blood flow to the region. This is followed by reperfusion when the effects of ET-1 wear off after several hours (Biernaskie et al., 2001). The reperfusion creates an ischemic penumbra (Weinstein et al., 2004; Gauberti et al., 2016), largely absent in PT stroke, corresponding to a region where neurons remain at risk but are salvageable (Heiss, 2012; Wetterling et al., 2016). PT strokes are induced by cortical photoactivation of a light-sensitive dye that is administered peripherally, resulting in singlet oxygen production, endothelial damage, platelet activation and aggregation, causing permanent occlusion of vessels in the irradiated region of the brain (Uzdensky, 2018). ET-1 and PT stroke models precisely target cortical regions relevant to cerebrovascular and behavioral recovery, are reproducible, and more closely mimic the size (on a proportional basis) of human strokes, with or without reperfusion. There is minimal edema associated with the ET-1 model (Schirrmacher et al., 2016) and lack of BBB disruption (Hughes et al., 2003), while PT stroke is associated with simultaneous cytotoxic edema due to cell death and vasogenic edema due to BBB disruption (Chen et al., 2007). This varies from the primarily cytotoxic edema seen initially in human stroke which is later followed by vasogenic edema (Provenzale et al., 2003). Furthermore, PT stroke corresponds with a strong immunogenic response characterized by increased infiltration of circulating leukocytes, as well as high levels of ROS and pro-inflammatory cytokines (Cotrina et al., 2017). Both PT and ET-1 are reproducible, convenient, and minimally invasive, however, they must be used accordingly regarding these considereations.

Perhaps the most accurate representation of ischemic stroke as seen in humans is the thromboembolic model of embolic stroke, whereby spontaneous or thrombin-induced clots of heterologous or autologous blood are injected into a cerebral artery. Alternatively, thrombin can be directly injected into the MCA or internal carotid artery to induce vascular occlusion. This accurately represents vascular occlusion most often seen in humans; however, the thrombi are mainly composed of polymerized fibrin, and therefore differ from thrombi in human patients that contain large amounts of both thrombin and erythrocytes (Duffy et al., 2019). Nevertheless, use of thrombolytic agents in this stroke model has the potential to mimic reperfusion following treatment that current stroke models do not as accurately represent (Fluri et al., 2015). Additionally, variability in clot size and stability results in variable infarct size and location. While thromboembolic stroke provides an accurate clinical representation of stroke in terms of edema, BBB breakdown, and inflammatory response, the inherent variability of the model requires large sample sizes to overcome this (Sommer, 2017).

In addition, the choice of anesthetic regimen is crucial when performing stroke surgery in rodents, as it can strongly influence CBF and stroke outcome, and may contribute to translational failure (O’Collins et al., 2006). For instance, isoflurane is a potent vasodilator with neuroprotective effects (Tsuda, 2010; Gaidhani et al., 2017; Jiang et al., 2017; Lu et al., 2017) via modulation of eNOS activity (Kehl et al., 2002; Krolikowski et al., 2006), which strongly confounds results. Ketamine/Xylazine (K/X) anesthesia affects baseline CBF to a lesser extent, but has also been shown to modulate eNOS (Chen et al., 2005). To circumvent these methodological obstacles, one should compare stroke outcomes in anesthetized versus awake mice when possible.

Overall, there is an urgent need to carefully refine experimental designs to prevent translational failure. In depth comparisons of the advantages and disadvantages of currently used stroke models and their applications in different areas of research has been reviewed elsewhere (Fluri et al., 2015; Sommer, 2017). Choosing the appropriate stroke model is essential to provide meaningful data and avoid translational failure.

### What the Future Holds for Cerebrovascular Stroke Research

Unfortunately, stroke research has suffered many setbacks, primarily due to a number of potential therapeutic candidates that have not delivered the expected benefits. As such, industry investment in the field dwindled owing to the perception of stroke research as a high-risk/low reward investment. Most negative results stemmed from failure of scientists to apply the information supplied by animal models to clinical trials. One compelling example, *N*-methyl-D-aspartate (NMDA) antagonists were only found to be neuroprotective when given to rats up to 90 min after blood vessel occlusion. However, in clinical trials patients were not given these drugs until 6 h later (Green and Shuaib, 2006). Despite these setbacks, researchers are continuously developing new methods and refining models, as well as investigating novel avenues of research that hold significant promise in improving stroke outcome (Silasi et al., 2015; Gouveia et al., 2017; Kannangara et al., 2018; Freitas-Andrade et al., 2019; Hill et al., 2020; Mendonca et al., 2020; Rayasam et al., 2020; Zhang et al., 2020). A greater appreciation for the role of physical rehabilitation and insight into the molecular mechanisms at play has led to a significant impact on the quality of life after stroke (Fang et al., 2019; McDonald et al., 2019; Sun and Zehr, 2019).

Novel molecules and new approaches focused on manipulating the cerebral vasculature to mitigate the effects of stroke are ongoing (Stanimirovic et al., 2018; Kanazawa et al., 2019). For example, Salvinorin A (derived from the ethnomedical plant Salvia divinorum), a selective kappa opioid receptor (KOR) agonist (Butelman and Kreek, 2015), has been shown to reduce cerebral vasospasm and alleviate brain injury after SAH via increasing expression of eNOS, and decreasing ET-1 concentration and AQP-4 protein expression (Sun et al., 2018). A recent study also showed that this drug can protect EC mitochondrial function following stroke (Dong et al., 2019). Remarkably, cutting-edge techniques, such as, single-cell RNA sequencing are unmasking the inner workings of ECs at an unprecedented level (Vanlandewijck et al., 2018; Munji et al., 2019; Kalucka et al., 2020; Kirst et al., 2020; Rohlenova et al., 2020). Finally, rigorous guidelines for effective translational research have been proposed, including the use of rodent models that are more representative of human strokes integrating comorbidities (Lapchak et al., 2013; Reeson et al., 2015). Given that the incidence of stroke increases with vascular diseases, animal models that incorporate comorbidities are critical in stroke research. A clinical study demonstrated that patients with chronic cerebral small vessel disease were associated with poor recruitment of collaterals in large vessel occlusion stroke (Lin et al., 2020). Another comorbidity, hypertension, is a modifiable risk factor for stroke. Hypertension is prevalent in the stroke population and is an important comorbidity to investigate (Cipolla et al., 2018). Hypertension promotes stroke through increased shear stress, endothelial cell dysfunction and large artery stiffness that transmits pulsatile flow to the microcirculation in the brain. Indeed, dysfunctional angiogenesis may occur in diabetic and/or hypertensive elderly patients in the recovering penumbra following stroke (Ergul et al., 2012).

While exciting new developments are in the pipeline, several lines of investigation indicate a significant impact lifestyle has on vascular health (Hakim, 2014, 2019) and particularly on brain angiogenesis and stroke outcome (Schmidt et al., 2013). A short interval of exercise prior to stroke was shown to improve functional outcomes by enhancing angiogenesis (Pianta et al., 2019). A possible mechanism of action was demonstrated to result from exercise-induced increase in VEGF expression via the lactate receptor HCAR1 in the brain (Morland et al., 2017). However, other mechanisms including growth factors or eNOS-dependent pathways have been reported (Geiseler and Morland, 2018).

Therefore, the scientific community must emphasize the importance of lifestyle in reducing the burden of stroke; we have the knowledge and responsibility to urge implementation of more extensive public health awareness and strategies to promote healthy vascular aging.

## Author Contributions

BL chose the theme of the review. MF-A, JR-N, and BL wrote the manuscript. All authors contributed to the article and approved the submitted version.

## Conflict of Interest

The authors declare that the research was conducted in the absence of any commercial or financial relationships that could be construed as a potential conflict of interest.
